# Analysis of Intervention Effect and Satisfaction of Holistic Nursing after Oral Tumor Resection

**DOI:** 10.1155/2022/3788605

**Published:** 2022-07-15

**Authors:** Lingling Qu, Yan Yin, Na Zhao, Yongmei Lv, Hangyong Xu

**Affiliations:** ^1^Rehabilitation Department, Yantaishan Hospital, Yantai 264000, China; ^2^Department of Infectious Diseases, Qingdao Eighth People's Hospital, Qingdao 266100, China; ^3^Department of Otorhinolaryngology, Zhangqiu District People's Hospital, Jinan 250200, China; ^4^Department of Pharmacy, Zhangqiu District People's Hospital, Jinan 250200, China; ^5^Department of Oral and Maxillofacial Surgery, Zhangqiu District People's Hospital, Jinan 250200, China

## Abstract

**Objective:**

To explore the intervention effect and satisfaction analysis of holistic nursing after oral tumor resection.

**Methods:**

A total of 70 oral tumor patients who underwent surgical treatment in our hospital from April 2020 to September 2021 were randomly divided into two groups, with 35 patients in each group. The control group was given basic oral care, the observation group was given overall oral care, and the actual effects of the two groups of care were compared, including the emotional status, compliance and nursing satisfaction, hospital stay and nursing quality scores, pain level, quality of life, and complications occurred.

**Results:**

After nursing, the patients in the observation group had good mood, higher compliance and nursing satisfaction, shorter hospital stay, higher nursing quality and quality of life scores, lower pain level, and lower incidence of complications, when compared with the control group.

**Conclusion:**

Holistic nursing has obvious effects on patients after oral tumor surgery, which can relieve patients' negative emotions, improve patients' compliance with treatment, improve their quality of life, and effectively reduce the degree of pain and the occurrence of complications, which is worthy of clinical promotion.

## 1. Introduction

Oral tumors are the most common malignant tumors of the head and neck, with a high incidence rate, accounting for 8.0% of systemic tumors [1–3]. In clinical medicine, surgical treatment is generally used as the way of treatment, but due to the complex surgical method, long operation time, and large postoperative wound, the internal self-cleaning effect of oral cavity is reduced to a certain extent, resulting in a high probability of bacterial infection. Once infection occurs, the patient's quality of life will be reduced, the wound will not heal well, and even the peripheral organs and tissues will be involved, seriously or even directly endangering life [4–6]. In addition, the postoperative facial damage leads to the accumulation of negative emotions such as depression and anxiety, which greatly affects the wound healing and postoperative recovery of patients. Therefore, a set of targeted and time-sensitive care plans is needed to reduce the negative emotions of patients and promote disease outcomes. In this study, 70 patients who underwent radical resection of oral tumors in our hospital were selected for nursing intervention, and the effects were satisfactory.

## 2. Materials and Methods

### 2.1. Basic Information

A total of 70 oral tumor patients who underwent surgical treatment in our hospital from April 2020 to September 2021 were selected, and the patients were randomly divided into the observation group (*n* = 35) and the control group (*n* = 35). There were 21 males and 14 females, ranging in age from 31 to 67 years old, with an average age of 44.5 ± 5.5 years, and the course of disease was 2.3 to 10.5 months, with an average of 5.3 ± 2.2 months; the control group consisted of 23 males and 12 females, aged 33 years old to 65 years old, average 45.5 ± 4.7 years old, disease duration 2.2 ~ 10.9 months, and average 5.4 ± 2.3 months. Inclusion criteria are as follows: patients were diagnosed with oral tumors according to clinical medical tests and meets surgical and oral tumor criteria [7], and the patients and their families gave informed consent to this study. Exclusion criteria are as follows: patients were diagnosed with mental illness or confusion and patients who did not cooperate with the treatment and care. There was no significant difference in the basic data of age, gender, and course of disease between the two groups, which was comparable. This study was approved by the ethics committee of Zhangqiu District People's Hospital (approval no. 2020-0632).

### 2.2. Nursing Methods

The patients in the control group received routine nursing guidance, including admission introduction, guided patient examination, close monitoring of the condition, basic ward nursing, and symptomatic intervention. The patients in the observation group carried out overall nursing intervention under routine guidance, including the following: ① postural care: for patients who are under general anesthesia and have not woken up after surgery, they are placed in a supine position, and their head is kept on the side; for patients with pedicled skin flaps, the head needs to be placed in the median position after surgery, and the supine immobilization is performed for 5-7 days to promote local blood circulation. ② Nutritional intervention: the next day after the operation, the patients were given nasal feeding, about 200 mL each time. It should be injected at a constant speed and nutritionally balanced. The lumen should be properly rinsed before and after the nasal feeding to reduce the occurrence of intestinal infection, the nasal feeding is changed to liquid food, and it is gradually transitioned to normal food [8]. ③ Negative pressure drainage and wound observation: doctor should closely observe the wound to determine whether there are problems such as oozing and swelling, check whether the dressing is damaged or not and whether the dressing is dry, and change the dressing once a day in the early postoperative period, and pay attention to keeping the wound clean and to observe whether the negative pressure drainage is unobstructed. Generally, the drainage volume in 24 hours should be >250 mL. If the drainage fluid is bright red and the amount is too large, it may be that the bleeding has not been completely stopped, and the doctor should be notified in time. ④ Eliminate the patient's saliva and sputum: after the operation, the patient's oral function is reduced, there is difficulty in swallowing, and the drooling is serious. One week after the operation, the patient's tongue is endangered. For example, the patient's tongue can only be extended halfway, and the contraction is difficult, and the internal oral cleaning cannot be carried out. All that needs to be done well is the propaganda work, informing the patient that saliva is beneficial for cleaning the inside of the mouth, moisturizing the throat and assisting the digestion and absorption of food materials, and swallowing the saliva in the mouth as much as possible. Adjust the pressure value and use a suction tube to suck out the saliva and sputum inside the mouth. ⑤ Cleaning: the doctor should clean with cotton wool moistened with silver ion mouthwash, in a gentle posture, wipe off sputum scabs and blood clots, and replace with 0.9% sodium chloride injection or silver ion mouthwash for cleaning. Patients with free tongue movement can instruct the patient to use their tongue. Massage the lingual side of the teeth in a certain direction, so that the lingual side of the teeth can be effectively cleaned, until the clear liquid is sucked out. The initial cleaning solution is generally more than 300 mL, and the other cleaning solution is preferably not more than 250 mL each time. It is cleaned twice a day, and patients with malignant tumors are cleaned three times a day. When cleaning, it should be noted that the cleaning solution directly cleans the mouth flap, and the cleaning tube should not touch the mouth flap, while rinsing and sucking, and the patient's tongue should be stirred at the same time [9]. ⑥ Strengthen the pain assessment of patients and do a good job in pain management. In this group of patients, the postoperative trauma was large, and the nerves in the oral cavity were rich and sensitive, but none of them were equipped with analgesic pumps to relieve pain. In knowledge-behavioral intervention therapy, informing patients that postoperative trauma is the main cause of pain, but negative emotions such as anxiety, depression, and irritability are powerful catalysts to increase pain and timely correct patients' bad cognition of pain, so as to avoid pain. The postoperative pain status of patients without tracheotomy was evaluated by the digital grading method. The resting pain was evaluated every 4 hours. Patients with 4 points received drug analgesia according to the doctor's advice. At the same time, patients were instructed to carry out regular breathing and muscle rhythmic exercise to eliminate patients' emotions and muscle tension, and timely and effective drug and physical analgesia methods were adopted. ⑦ Do a good job of psychological care to reduce negative emotions. Due to the special anatomy, oral tumor patients may have different degrees of facial disfigurement or deformity, functional impairment, and even death risk after surgery, which can easily lead to different degrees of mental and psychological disorders in patients after surgery, especially depression, anxiety, and fear. Other negative emotions are more prevalent and severe, and these negative emotions have a serious impact on postoperative recovery and patients' quality of life. Performing regular relaxation training after surgery, instructing the patient to relax the muscles of the whole body, and cooperating with deep breathing, instructing the patient to perform imagery imagination after completing the relaxation training, image pleasant scenes, and beautiful natural landscapes, and transferring postoperative pain such as dry mouth were done. Due to the temporary difficulty in opening the mouth and language dysfunction after the patient, our department uses a writing board to communicate with the patient in a timely manner. Communicating with patients through some simple gestures, shaking their heads, nodding, and other body language were also done.

### 2.3. Observation Indicators

The Hamilton Depression Scale (HAMD) and Hamilton Anxiety Scale (HAMA) were referred to evaluate the emotional status of the two groups at different nursing stages. The lower the score, the more significant the improvement of anxiety and depression were [10].

The self-made nursing questionnaire was used to investigate the compliance, nursing satisfaction, and nursing quality scores of the two groups.

The incidence of complications such as electrocution syndrome, bleeding, infection, and vascular crisis was counted.

The Visual Analogue Scale (VAS) for rating [11] was used to investigate the pain level of patients, with 10 points out of 10, and the lower the score, the less pain and the better the nursing effect.

The quality of life index evaluation scale [12] (Quality of Life Questionnare-Core 30 (QLQ-C30)) was used to evaluate the indicators of quality of life for patients.

### 2.4. Data Analysis Methods

The counting and measurement data of this study were input into the Statistical Products and Services Solutions 20.0 (Statistical Products and Services Solutions 20.0, SPSS 20.0, IBM, NY, USA) program was used for processing. Specifically, the chi-square and *t*-tests were completed. The output of the chi-square test results were displayed as (%), *t*-test results are displayed in the form of *x* ± *s*, and *p* < 0.05 indicates that the data difference is statistically significant.

## 3. Results

### 3.1. Analysis of Emotional Status in Different Nursing Stages after Surgery

At the end of the operation, there was no significant difference in HAMA and HAMD scores between the two groups. 1 d, 5 d, and discharge after the operation, the HAMA and HAMD scores of the two groups were lower than those at the end of the operation, and the scores between the two groups were lower than those at the end of the operation (Figure 1).

### 3.2. Comparison of Patient Compliance and Nursing Satisfaction between the Two Groups

The overall compliance of the observation group was 100%, which was significantly higher than that of the control group (80%). The nursing satisfaction of the observation group was 97.14%, which was significantly higher than that of the control group (71.43%) (Tables 1 and 2).

### 3.3. Comparison of Hospital Stay and Nursing Quality Scores between the Two Groups

There were statistically significant differences between the two groups in terms of hospital stay, basic nursing score, safety nursing score, disinfection nursing score, and ward nursing score (Table 3).

### 3.4. Comparison of Pain Levels between the Two Groups

There was no significant difference in the VAS score between the two groups at the end of the operation, and the VAS score gradually decreased with the increase of the end of the operation time (Figure 2).

### 3.5. Comparison of Quality of Life before and after Nursing in the Two Groups

Before nursing, there was no significant difference in the indicators of quality of life between the two groups. After nursing, the scores of physical function, role function, emotional function, cognitive function, and social function in the two groups were all increased, and the difference between the observation group and the control group was statistically significant. The scores of insomnia, fatigue, loss of appetite, diarrhea, and nausea and vomiting were obviously decreased (Table 4).

### 3.6. Comparison of the Incidence of Complications between the Two Groups

There were 1 case, 2 cases, 1 case, and 3 cases of electrical resection syndrome, hemorrhage, infection, and vascular crisis in the observation group and 7 cases, 9 cases, 6 cases, and 11 cases of electrical resection syndrome, hemorrhage, infection and vascular crisis occurred in the control group, respectively (Figure 3).

## 4. Discussion

According to statistics, oral tumors account for nearly 8% of human tumors [13, 14]. Due to the poor efficacy of conservative treatment, surgical treatment is currently recommended for diagnosed oral tumors [15]. However, the anatomical structure of the oral cavity is relatively complex, and the lesion site is relatively special. Tissue defects occur under various trauma or surgical treatment conditions. The patient's resistance and oral self-cleaning ability decline. The imbalance of the proportion of the group is very prone to local infection and even the occurrence of complications due to infection, resulting in a worse prognosis [16]. This makes patients generally have a heavy psychological and spiritual burden. Effective nursing interventions are very important. Some data show that [17–19] effective nursing intervention after oral tumor surgery has a significant effect on improving prognosis and improving the quality of life of patients.

Holistic care is one of the important modes of care and an intensification of routine care [20, 21]. It can fully combine the patient's disease characteristics and physical and mental conditions and use psychological education, postural care, nutritional intervention, and other measures to provide systematic services and guidance for patients from various aspects such as psychology, behavioral cognition, diet, and posture. It can not only ensure the actual effect of oral care but also achieve the comfort of patients, making oral care develop in a safer, more reasonable, more professional, and more personalized direction. At present, the application effect of holistic nursing in international clinical practice has been widely recognized, and its development in oral tumor patients has also been proved to have good effects such as reducing the occurrence of complications and promoting patient recovery [22–25]. This study showed that the HAMA and HAMD evaluation scores of the observation group were significantly lower than those of the control group after this model intervention. The reason is that the overall nursing care used in this study includes psychological nursing. Through the professional relaxation training of medical staff and the timely detection and processing of patients' inappropriate emotions, the patients in the observation group have better emotions than the control group, so the degree of cooperation and nursing satisfaction are higher. Our nursing plan also strengthens pain care and cleaning care for patients, so the results of this study show that the nursing quality score of the observation group is significantly higher than that of the control group, and the incidence of complications is significantly lower than that of the control group, thereby improving the overall quality of life of patients.

## 5. Conclusion

To sum up, the overall nursing intervention for patients after oral tumor surgery is effective, which can significantly reduce the patient's emotional burden, reduce the patient's pain level, effectively improve the quality of nursing services, reduce the risk of complications, and improve the quality of life. It can improve patients' recognition of nursing work and can be used as an excellent solution for clinical nursing, which is worthy of recommendation.

## Figures and Tables

**Figure 1:** Emotional status of the two groups after surgery in different nursing stages. (a) The HAMA score of the observation group decreased gradually at the end of the surgery, 1 d and 5 d after the surgery, and at discharge. (b) The HAMA score of the control group at the end of the surgery, the surgery after 1 d and 5 d, it gradually decreased at discharge. (c) The HAMD score of the observation group decreased gradually at the end of the operation, 1 d and 5 d after surgery, and gradually decreased at discharge. (d) The HAMD score of the control group was decreased after surgery at the end, 1 d, and 5 d postoperatively and gradually decreased at discharge. ^∗^*p* < 0.01, vs. end of operation.

**Figure 2:** Comparison of pain levels between the two groups. ^∗^*p* < 0.01 vs. the control group.

**Figure 3:** Comparison of the incidence of complications.  ^∗^*p* < 0.01 vs. the control group.

**Table 1:** Comparison of nursing compliance between the two groups (*n* (%)).

Group	*n*	Good	General	Poor	Overall compliance
Observation group	35	26 (74.29)	9 (25.71)	0 (0.00)	35 (100.00)
Control group	35	17 (48.57)	11 (31.43)	7 (2.00)	28 (80.00)
*X* ^2^					9.084
*p*					0.011

**Table 2:** Comparison of nursing satisfaction between the two groups (*n* (%)).

Group	*n*	Very satisfied	General	Dissatisfied	Overall satisfaction
Observation group	35	23 (65.71)	11 (31.43)	1 (2.86)	34 (97.14)
Control group	35	12 (34.29)	13 (37.14)	10 (28.57)	25 (71.43)
*X* ^2^					10.987
*p*					0.004

^∗^ *p* < 0.01 vs. the control group.

**Table 3:** Comparison of hospital stay and nursing quality score (*x* ± *s*).

Group	*n*	Hospital stay (d)	Quality of care			
			Basic care	Safe care	Disinfection care	Ward Care
Observation group	35	8.74 ± 1.44	94.17 ± 2.81	96.09 ± 2.23	97.14 ± 1.61	95.17 ± 2.24
Control group	35	12.00 ± 2.70	79.94 ± 4.08	81.89 ± 3.46	81.09 ± 2.89	83.49 ± 3.02
*t*		6.294	16.99	20.41	28.68	18.37
*p*		< 0.001	< 0.001	< 0.001	< 0.001	< 0.001

^∗^ *p* < 0.01 vs. the control group.

**Table 4:** Comparison of quality of life before and after nursing (*x* ± *s*).

Group	*n*	Nursing time	Physical function	Role function	Emotional function	Cognitive function	Social function
Observation group	35	Before nursing	51.83 ± 8.56	55.54 ± 9.86	49.51 ± 12.07	60.89 ± 6.60	58.71 ± 10.70
		After nursing	78.54 ± 10.71	87.00 ± 5.75	88.00 ± 5.29	81.09 ± 8.55	76.71 ± 10.93
Control group	35	Before nursing	54.20 ± 7.01	54.74 ± 8.59	51.49 ± 13.53	54.00 ± 7.75	59.54 ± 9.86
		After nursing	63.29 ± 11.70	74.29 ± 7.78	70.20 ± 7.01	60.54 ± 9.86	68.09 ± 8.55
*t*1			11.53	16.31	17.27	11.07	6.962
*p*1			< 0.001	< 0.001	< 0.001	< 0.001	< 0.001
*t*2			3.940	9.979	7.264	3.087	3.872
*p*2			< 0.001	< 0.001	< 0.001	0.003	< 0.001
*t*3			5.689	7.779	11.99	9.312	3.679
*p*3			< 0.001	< 0.001	< 0.001	< 0.001	0.001
Group	*n*	Nursing time	Insomnia	Tired	Anorexia	Diarrhea	Feel sick and vomit
Observation group	35	Before nursing	55.20 ± 12.05	53.31 ± 7.45	47.14 ± 7.75	42.69 ± 5.76	35.09 ± 10.79
		After nursing	20.57 ± 7.82	21.97 ± 6.57	17.14 ± 5.10	24.77 ± 4.70	7.49 ± 2.55
Control group	35	Before nursing	48.49 ± 7.39	52.31 ± 5.76	49.26 ± 6.34	45.00 ± 5.29	32.86 ± 10.67
		After nursing	38.00 ± 6.33	29.40 ± 7.05	31.37 ± 5.82	35.71 ± 7.78	15.43 ± 4.02
*t*1			14.27	18.67	19.12	14.25	14.73
*p*1			< 0.001	< 0.001	< 0.001	< 0.001	< 0.001
*t*2			6.378	14.89	12.29	5.893	9.044
*p*2			< 0.001	< 0.001	< 0.001	< 0.001	< 0.001
*t*3			10.25	4.562	10.88	7.125	9.879
*p*3			< 0.001	< 0.001	< 0.001	< 0.001	< 0.001

Note: *t*1, *p*1 represent the comparison before and after nursing in the observation group; *t*2, *p*2 represent the comparison before and after nursing in the control group; *t*3, *p*3 represent the comparison between the observation group and the control group after nursing. ^∗^*p* < 0.01 vs. the control group.

## Data Availability

The datasets used and/or analyzed during the present study are available from the corresponding author on reasonable request.
